# Repeatability and Image Quality of IDEAL-IQ in Human Lumbar Vertebrae for Fat and Iron Quantification across Acquisition Parameters

**DOI:** 10.1155/2022/2229160

**Published:** 2022-06-09

**Authors:** Ben Shan, Haiyan Ding, Qianzao Lin, Xiaohua Zuo, Lili Lin, Dongyang Yu, Chunhong Hu

**Affiliations:** ^1^Department of Radiology, The First Affiliated Hospital of Soochow University, 188 Shizi Street, Suzhou 215006, China; ^2^Department of Radiology, The Affiliated Huai'an Hospital of Xuzhou Medical University, 62 South Huaihai Road, Huai'an 223001, China; ^3^Department of Radiology, Huai'an Fifth People's Hospital, 1 East Huaihe Road, Huai'an 223001, China; ^4^Department of Pain Management, The Affiliated Huai'an Hospital of Xuzhou Medical University, 62 South Huaihai Road, Huai'an 223001, China; ^5^The First Clinical Medical College, Gansu University of Chinese Medicine, 35 East Dingxi Road, Lanzhou 730000, China

## Abstract

Echo asymmetry and least square estimation-IQ (IDEAL-IQ) were used to quantify fat and iron to verify the effects of collection parameters on repeatability and image quality of water and fat in human vertebral body. Six IDEAL-IQ sequences were used to scan 48 healthy adult women. Reproducibility of fat and iron quantification and image quality were assessed for six IDEAL-IQ sequences. The results showed that the correlation index (0.987, 0.721) of FF and R2∗ between scans of sequence 2 was higher than that of other sequences, and the consistency of fat quantification was better than that of iron (0.860 vs. 0.579) (*P* < 0.001). Sequence 2 had the highest image quality score (4.9) and the lowest CV score (9.2%). In the FF figure, SNR (18.8) and CNR (17.8 ± 6.4) were the highest, while CV was the lowest (36.7%, 36.1%). In the R2∗ figure, sequence 3 had the highest SNR (21.8) and CNR (20.5), but its CV (51.8% and 56.1%) was significantly higher than that of sequence 2. The occurrence of fat-water exchange (FWS) was lowest in sequence 2 and sequence 4 (0, *N* = 96). In conclusion, the fat quantification of IDEAL-IQ was robust to the changes of collection parameters, and section thickness (ST) had a certain effect on maintaining good repeatability of R2∗ quantification. The higher the ST was, the better the image quality of FF and R2∗ was maintained and stable and the less the occurrence of FWS.

## 1. Introduction

In recent decades, with the development of medical imaging equipment and the innovation of various imaging technologies, imaging biomarkers have attracted more and more attention from researchers around the world, including quantitative and qualitative [1]. Many studies suggested that magnetic resonance imaging (MRI) has the advantages of multiparameter imaging, no radiation damage, and good soft tissue contrast, so it has been widely used in related fields [2]. However, the signal intensity of conventional MRI is mainly composed of water and fat, so the content or proportion of water and fat in human tissues can be accurately quantified. Vertebral body fat and water content is normal or is not very important to people's daily activities. When there is vertebral body fat deposition, the limited amount of it will not cause significant impact. However, the excessive deposition may produce repeated lumbar pain and oppressive nerve symptom such as intermittent claudication, lower limb weakness, and similar symptoms of intervertebral disc herniation. Therefore, MRI can provide a new idea for the study of vertebral diseases.

Studies indicated that a commercial volumetric MRI technique, the iterative factory-IQ (IDEAL-IQ) of water and fat with echo asymmetry and least-square estimation, can quantify fat and iron in target tissues from a single scan with fat fraction (FF) and R2∗ plots [3]. As the robustness, precision, repeatability, and reproducibility of this technique have been elaborated [4–7], it has gradually become a hotspot in relevant directions in recent years. There are some investigators started trying to use it to quantify the FF and R2∗ values of the vertebrae and found that the bone marrow fat content of the lumbar spine correlated with adjacent disc degeneration [8], the bone marrow fat content and microvascular permeability of the vertebrae in diabetic rabbits [9], and vertebral fat quantitation were robust to changes in R2∗ [10].

As a proton density imaging technique, fat quantification by IDEAL-IQ should be free from scanner setting and acquisition parameters [11]. Still, Rajlawot et al. most recently reported that the flip angle (FA) could affect the measurement of hepatic FF as well as the image quality of IDEAL-IQ [12]. We, therefore, proposed the hypothesis that the acquisition parameters might affect its repeatability and image quality in vertebrae. Good repeatability and image quality are essential traits and prerequisites for a reliable imaging biomarker, especially in radiomic study [13]. To our knowledge, the manufacturer has not provided standardized parameters for the vertebral application, and previous studies have shown significant variations in acquisition parameters, both in the liver and vertebrae. Hence, this study was committed to verifying the impact of acquisition parameters on the repeatability and image quality of IDEAL-IQ in human vertebrae, which will help to optimize and standardize this technique and maintain the homogeneity of the relevant research.

## 2. Materials and Methods

### 2.1. Study Population

Forty-eight adult women volunteered to participate in this study. The average age was 51.9 ± 11.8 years (from 26 to 79 years), the average weight was 62.1 ± 8.8 kg (from 45 to 89 kg), and the average height was 158.8 ± 4.7 cm (from 145 to 168 cm). None of the participants was clinically diagnosed with any major illness in the physical examination within 1 month or had a history of drug or alcohol abuse. Male volunteers were not included to avoid the potential impact of gender on bone marrow fat or iron content in the vertebral body. All volunteers signed informed consent forms, and this experiment had been approved by ethics committee of hospital.

### 2.2. Bone Mineral Density Examination

All subjects underwent dual energy X-ray absorptiometry bone mineral density (BMD) scan using a Lunar iDXA scanner (GE Healthcare, Madison, WI, USA) with the patient lying flat on the examination bed in the supine position, and the scan range included the 1st to 4th lumbar vertebra.

### 2.3. IDEAL-IQ Sequences

A serial IDEAL-IQ sequences for lumbar vertebrae (L1-5) were designed in this study using a GE Discovery 750w 3.0T scanner (GE Healthcare, Florence, SC, USA) with an eight-channel CTL spine coil. Basic acquisition parameters were as follows: scan plane = sagittal, FOV =32 × 32 cm, frequency direction = A/P, number of shots =2, TE = minimum full (1.1-12.2 ms), TR = auto (9.1-20.1 ms), Locs per slab =8, and matrix =160 × 160. Other detailed parameters for each sequence are shown in Table 1. All of 48 volunteers underwent the serial IDEAL-IQ scans twice consecutively by two independent radiographers with reposition.

### 2.4. Image Quality Assessment and Data Measurement

A qualitative visual assessment of the overall image quality for each IDEAL-IQ sequence was performed using a five-point scoring scale on FF and R2∗ maps. Five corresponded to excellent image quality; the border and internal structure of vertebrae could be displayed perfectly (Figures 1(a) and 1(b)). Four corresponded to good image quality, with few artifacts. Three corresponded to average image quality, with more artifacts or blurred areas. Two corresponded to poor image quality, with many artifacts or blurred areas; some area of the border or internal structure could not be clearly displayed. One corresponded to inferior image quality; most site of the border or internal structure could hardly be distinguished (Figures 1(c) and 1(d)).

Data measurement was performed using Advanced Workstation 4.6 (AW4.6, GE Healthcare). First, a region of interest (ROI) was manually drawn on 3rd lumbar spine (L3) for FF or R2∗ measurement, along the outer border of the vertebral body on the most central slice to encompass maximum bone marrow area while avoiding confounding structures such as the bony cortex and blood vessel clearly shown (Figure 1(a), blue ROI). Then, another ROI was drawn on the same slice in the spinal canal posterior to L3 to encompass as much cerebrospinal fluid as possible while avoiding confounding structures such as the osteophyte, nerve, and ligament clearly showed (Figure 1(a), red ROI). The FF or R2∗ value of the L3 vertebral body represented the target signal intensity (SI); the corresponding value of cerebrospinal fluid (CSF) represented the contrast (C); the standard deviation (SD) of CSF represented the noise (N). Signal to noise ratio (SNR) and contrast to noise ratio (CNR) were calculated using the following formulas:

(1) $$\begin{array}{c} \text{SNR}=\left|\text{SI}/N\right|, \end{array}$$

(2) $$\begin{array}{c} \text{CNR}=\left(\text{SI}-C\right)/N. \end{array}$$

All image scores and drawings of ROIs were determined by an experienced radiologist and an experienced radiographer together to reduce subjective bias, both of which were blinded to volunteers' information and the detailed parameters.

### 2.5. Statistical Analysis

Statistical analyses were performed using MedCalc Statistical Software version 19.3.1 (MedCalc Software Ltd, Ostend, Belgium). The quantitative data in accordance with normal distribution were expressed by mean ± SD, and those in disagreement were expressed by mean (range). Intraclass correlation coefficient (ICC) with two-way mixed model and absolute agreement type and the Bland-Altman plots were performed to evaluate the repeatability of FF and R2∗ measurements. Interscan ICC was committed between the first scan and the second scan, and Intersequence ICC was committed between sequences 1 and 6 with pooled data. *P* < 0.05 was considered to indicate a statistically significant difference.

## 3. Results

### 3.1. Participants

A total of 48 healthy adult women participated in this study, with an average age of 51.9 ± 11.8 years (from 26 to 79). Other major clinical and BMD indicators of L3 are shown in Table 2.

### 3.2. Fat Fraction and R2∗ Measurements and Interscan and Intersequence Agreement Analyses

The FF and R2∗ values of L3 of the two scans and the pooled data were measured and calculated, and ICCs of interscan and intersequence were analyzed, as shown in Table 3.

For the measurement of FF, good agreements of interscan and intersequence could be seen; but for R2∗ measurement, it could only be seen between two repeated scans of sequence 2 (with ICC > 0.7). Sequence 2 had the best consistency of repeated scans in both fat and iron quantification. The Bland-Altman plots of each sequence for FF and R2∗ quantification were shown in Figure 2 (Online Resource).

### 3.3. Image Quality Assessment

For each independent sequence, the FF and R2∗ maps had relatively consistent visual image quality, so the image quality score of the FF map was used to represent the overall image quality in this study. The overall image quality score, SNR, and CNR of FF and R2∗ maps and their coefficients of variation (CVs) calculated using pooled data are demonstrated in Table 4.

The subjective evaluation showed that sequence 2 had the highest image quality score and the lowest CV, suggesting that its overall visual image quality was the best and the most stable. For FF maps, the highest SNR and CNR with the lowest CV could also be found in sequence 2, indicating that its image quality is the highest and the most stable. However, in R2∗ maps, sequence 2 had the second highest SNR and CNR with the lowest CV; the SNR and CNR of sequence 3 were the highest, but their CVs were significantly higher than that of sequence 2, suggesting that the image quality was not much stable. In general, the visual image quality score, SNR, CNR, and the CVs of sequence 5 were all the worst.

### 3.4. Fat-Water Swap

In this study, a fat-water swap (FWS) phenomenon (Figures 1(e) and 1(g)) could be observed from time to time, in which other components such as blood or cerebrospinal fluid were replaced by fat in FF maps, in whole or in part.  Table 5 demonstrates the frequency of FWS in different sequences in a total of 96 independent serial scans.

The FWS was not observed in sequences 2 and 4, and it was most common in sequence 3, followed by sequences 6, 1, and 5. We also found that the correct FF map could be obtained for each sequence by repeated scan free of repositioning.

## 4. Discussion

MRI is an ideal and reliable way for fat quantification at present, which avoids radiation exposure by dual energy X-ray or quantitative CT. At the same time, ultrasonography can carry out direct and complete fat quantification [14]. On the other hand, all current noninvasive iron quantification methods are almost MRI-dependent. Nowadays, magnetic resonance spectroscopy (MRS) is still regarded as the gold standard for noninvasive fat and iron quantification, but it also has some disadvantages. First, the time of MRS signal acquisition is too long, which means that it requires much more cooperation from the patients, including holding breath and tolerating noise. Second, it can only perform single-site sampling instead of volumetric scanning; that is, sampling bias. Finally, the technical precision of MRS may need to be reconsidered because of the lack of sufficiently high spectral resolution at clinical field strengths, resulting in difficulty in completely distinguishing the water and fat peaks on fat quantification [11, 15]. Therefore, the ideal IDEAL-IQ requires full consideration and correction of confounding factors. Multiecho signal acquisition and iterative least square decomposition algorithm can not only calculate T2∗ fitting but also conducive to the complete decomposition of water and fat signals as well as maintain the homogeneity of the magnetic field; tiny FA can largely overcome T1 bias; multipeak fat model fitting can reasonably simulate the complex composition of fat in the human body; resulting in a robust and accurate fat quantification [10]. These techniques are also effective for R2∗, in other word, iron quantification [6]. Therefore, theoretically, IDEAL-IQ should outperform conventional MRI techniques in fat and iron quantification, such as two-point Dixon and MRS [16, 17].

For this study, all subjects were scanned twice independently, and then, the data measurement and image scoring were performed jointly by a radiologist and a radiographer, because we thought this study protocol was more representative of the repeatability of imaging technology and appropriate for minimizing subjective bias. Based on this protocol, we found a potential instability that may exist with R2∗ quantification which was different from a previous study [16], and this should not be mainly due to change in a research setting but the acquisition parameters. The basic scanning protocol (sequence 1) was designed to pursue the minimum available slice thickness (ST) of 2.7 mm as well as suitable acquisition time in this experimental model, as small ST was advantageous for reducing partial volume effect and obtaining higher spatial resolution which may be critical for some advanced studies [13, 18], and excessive acquisition time was unfavorable for clinical application. Based on this, several parameters that might influence the outcome were adjusted, one for each sequence.

Increasing the ST allowed obtaining more signal sources, reducing the image noise [13], weakening the impact of field heterogeneity [19], and increasing the T2∗ fitting [20], so sequence 2 was shown to have the best quantitative repeatability (especially in R2∗ quantification) as well as overall image quality and stability. Mi et al. also found that the repeatability of radiomic features was better with increasing ST [21], which was consistent with our study. The change resulting from increasing the number of excitation (NEX) could be explained by the same theory, but this change was less pronounced than in ST. Increasing the bandwidth (BW) led to an increase in image noise, which was opposite to the echo train length (ETL) [22]. The increased BW and ETL in the IDEAL-IQ sequence were accompanied by a significantly longer repetition time, which would make the SNR of CSF significantly increased [23]. Therefore, sequence 6 showed a mild decrease in both subjective and objective image quality, and sequence 3 showed a significant elevation of objective image quality but not a subjective one, which was consistent with the previous studies [22, 23]. Increasing FA resulted in a significantly accentuated T1 bias, which was critical for IDEAL-IQ and was not compensated by any other factor, ultimately led to both the worst subjective and objective image quality.

Regarding the FWS, which is closely related to the ambiguity of field map estimation during fat-water separation, has gained the attention of many researchers in recent years [24]. In the present study, for the first time, we found the possible potential influence of acquisition parameters on this phenomenon. It could be attenuated by increasing ST and NEX, possibly due to both increased signal acquisition and reduced noise bias, which closely correlated with field map estimation [25] and required a larger sample size for validation. As mentioned above, a longer repetition time accompanied by increased ETL and BW would result in obviously elevated SNR in cerebrospinal fluid but insignificant in spine marrow fat [23], generating susceptibility artifact, which would cause decomposition error and eventually the occurrence of FWS [24, 26].

Rajlawot et al. found that an increase in FA from 3 to 8 and 9 degrees helped improve SNR and CNR for liver fat quantification [12], which was different from the conclusion of our study and might be based on the following reasons. First, our study setting was the spine, and the contrast was cerebrospinal fluid, not liver and muscle. Second, we employed FF and R2∗ maps for direct analysis, rather than the water map. Third, our study was based on a 2.7 mm ST, whereas their conclusions were drawn at 8 mm. We should also recognize that the target and contrast areas might be affected by the different degree of noise at the same time, so SNR and CNR in this study did not fully reflect the actual image quality, and it was equally important to assess the visual image quality.

We recognized that the present study also had some flaws. First, in the early stage of the study, we found that an ST of 4 mm was similarly accompanied by a high incidence of the FWS and poor image quality, so we directly adopted the ST of 8 mm, disregarding 5-7 mm. Second, because of the characteristic of the FF map [22], it was not suitable for selecting muscle or air in vitro as the contrast, so we tentatively adopted the CSF. There was a certain subjective bias in both the delineation of contrast ROIs and the judgment of confounding structures in this case. Third, we only demonstrated FF and R2∗ of L3, as well as SNR and CNR, because we found that the results of other vertebrae were roughly similar, and L3 was well representative.

## 5. Conclusion

In this study, echo asymmetry and least square estimator-IQ (IDEAL-IQ) were used to quantify fat and iron to verify the effects of collection parameters on the repeatability and image quality of water and fat in human vertebral body. It was found that the fat quantification of IDEAL-IQ was robust to the changes of collection parameters, and section thickness (ST) had a certain effect on maintaining good repeatability of R2∗ quantification. The higher ST was, the better the image quality of FF and R2∗ was maintained and stable and the less the occurrence of FWS. However, the sample size and scope of this study are limited, and the representativeness is insufficient, which requires further investigation. Currently, although the influence of acquisition parameters has not received enough attention in the application, the application of IDEAL-IQ technology in the field of vertebrae has shown broad prospects and is worthy of expectation.

## Figures and Tables

**Figure 1:** Image quality assessment and ROI delineation strategy. (a) FF and (b) (R2∗), 77 years old, sequence 2, the border and internal structure of vertebrae were perfectly displayed, scored 5 points. The schematic ROI of L3 was marked in blue and the contrast ROI in red. (c) FF and (d) R2∗, 33 years, sequence 5, most site of the border and internal structure of vertebrae could hardly be distinguished, scored 1 point. (e) FF and (f) R2∗, 46 years, sequence 3, a complete fat-water swap could be observed, with all regions of the FF map being disturbed. (g) FF and (h) R2∗, 53 years, sequence 6, a partial fat-water swap was observed, with some area of the FF map being disturbed.

**Figure 2:** The Bland-Altman plots of each sequence for FF and R2∗ quantification (Online Resource). (a)–(f) were plots for FF quantification, g-l for R2∗, of sequence 1-6, respectively. Sequence 2 showed the best agreement for both FF and R2∗ quantification.

**Table 1:** Supplementary detailed parameters of each IDEAL-IQ sequence.

	Sequence 1	Sequence 2	Sequence 3	Sequence 4	Sequence 5	Sequence 6
Slice thickness (mm)	2.7	***8***	2.7	2.7	2.7	2.7
Echo train length	3	3	***6***	3	3	3
NEX	1	1	1	***2***	1	1
Flip angle (°)	3	3	3	3	***5***	3
Bandwidth (Hz)	83.33	83.33	83.33	83.33	83.33	***166.67***
Scan time (s)	31	***24***	***52***	***62***	31	***42***

Bold italics: each adjusted parameter per sequence relative to sequence 1 was marked by bold italics.

**Table 2:** Main characteristics of 48 participants.

	Average	Range
Age (years)	51.9 ± 11.8	26~79
Weight (kg)	62.1 ± 8.8	45~89
Height (cm)	158.8 ± 4.7	145~168
BMI (kg/m^2^)	24.6 ± 3.6	17.6~35.6
BMD (g/cm^2^)	0.986 ± 0.199	0.537~1.452
*Z*	0.5 ± 1.2	-1.8~4.3
*T*	−0.4 ± 1.7	-4.3~4.4

BMI = body mass index; BMD = bone mineral density.

**Table 3:** Fat fraction and R2∗ measurements and interscan and intersequence agreement analyses.

		Sequence 1	Sequence 2	Sequence 3	Sequence 4	Sequence 5	Sequence 6
FF	1^st^ scan	46.2 ± 12.9%	45.7 ± 12.9%	48.3 ± 16.8%	46.1 ± 12.9%	46.2 ± 11.9%	46.3 ± 12.9%
	2^nd^ scan	46.2 ± 13.3%	45.6 ± 12.7%	48.5 ± 16.8%	46.1 ± 13.2%	45.0 ± 11.0%	46.2 ± 13.4%
	Pooled	46.2 ± 13.1%	45.7 ± 12.8%	48.4 ± 15.6%	46.1 ± 12.9%	45.6 ± 11.3%	46.2 ± 12.8%
	Interscan ICC	0.976^∗^	0.987^∗^	0.725^∗^	0.961^∗^	0.952^∗^	0.898^∗^
	Intersequence ICC	0.860^∗^					
R2∗	1^st^ scan	154.6 ± 38.2	151.5 ± 33.7	155.0 ± 32.1	158.7 ± 33.1	144.1 ± 23.9	154.5 ± 36.6
	2^nd^ scan	155.2 ± 30.1	148.2 ± 31.3	153.5 ± 34.2	158.5 ± 30.8	143.0 ± 32.3	161.6 ± 53.6
	Pooled	154.9 ± 30.7	149.9 ± 30.2	154.3 ± 27.8	158.6 ± 29.1	143.6 ± 24.1	158.1 ± 40.7
	Interscan ICC	0.597^∗^	0.721^∗^	0.412^#^	0.664^∗^	0.447^∗^	0.577^∗^
	Intersequence ICC	0.579^∗^					

FF = fat fraction; ICC = intraclass correlation coefficient. ^∗^*P* < 0.001 and ^#^*P* < 0.01.

**Table 4:** Image quality assessment of each sequence.

		Sequence 1	Sequence 2	Sequence 3	Sequence 4	Sequence 5	Sequence 6
Overall	Image quality score	3.4 (2-5)	4.9 (3-5)	3.5 (1-5)	3.8 (2-5)	1.8 (1-4)	2.7 (2-5)
	CV	17.0%	9.2%	21.7%	13.7%	33.5%	23.3%
FF	SNR	11.9 (5.2-27.0)	18.8 (7.0-34.3)	17.7 (6.3-44.3)	14.5 (6.8-34.0)	7.7 (3.9-19.0)	10.9 (5.0-24.7)
	CV	38.3%	36.7%	49.2%	39.4%	42.8%	39.3%
	CNR	10.9 (4.8-25.8)	17.8 ± 6.4	14.6 ± 6.8	13.6 ± 5.3	6.6 ± 3.0	9.5 ± 4.1
	CV	36.9%	36.1%	46.6%	39.2%	46.0%	43.0%
R2∗	SNR	13.0 (6.5-76.3)	16.3 (9.2-27.1)	21.8 (8.4-79.8)	13.8 ± 3.8	6.9 (3.0-43.7)	10.1 (4.6-23.4)
	CV	76.8%	26.1%	51.8%	27.5%	84.3%	35.3%
	CNR	12.1 (5.6-76.0)	14.8 ± 4.2	20.5 (7.1-79.5)	12.7 ± 3.9	6.1 (2.2-43.2)	9.2 (3.4-22.7)
	CV	83.5%	28.4%	56.1%	30.8%	96.1%	39.1%

SNR = signal to noise ratio; CNR = contrast to noise ratio; CV = coefficient of variation.

**Table 5:** Frequency of fat-water swap in different sequences.

	Sequence 1	Sequence 2	Sequence 3	Sequence 4	Sequence 5	Sequence 6
Fat-water swap	2	0	8	0	1	4

## Data Availability

This program was registered at Chinese Clinical Trial Registry (http://www.chictr.org.cn, Registration Number: ChiCTR2000032115). We were committed to raw data release after the end of the program.

## References

[1] Vamvakas A., Williams S. C., Theodorou K. (2019). Imaging biomarker analysis of advanced multiparametric MRI for glioma grading. *Physica Medica*.

[2] Yoneda N., Matsui O., Kobayashi S. (2019). Current status of imaging biomarkers predicting the biological nature of hepatocellular carcinoma. *Japanese Journal of Radiology*.

[3] Karcaaltincaba M., Idilman I., Celik A. (2011). Focal sparing of iron and fat in liver tissue in patients with hemosiderosis: diagnosis with combination of R2∗ relaxometry and proton density fat fraction calculation by MRI. *Diagnostic and Interventional Radiology*.

[4] Schmeel F. C., Vomweg T., Träber F. (2019). Proton density fat fraction MRI of vertebral bone marrow: accuracy, repeatability, and reproducibility among readers, field strengths, and imaging platforms. *Journal of Magnetic Resonance Imaging*.

[5] Kim H. J., Cho H. J., Kim B. (2019). Accuracy and precision of proton density fat fraction measurement across field strengths and scan intervals: a phantom and human study. *Journal of Magnetic Resonance Imaging*.

[6] Rostoker G., Laroudie M., Blanc R. (2019). Histological scores validate the accuracy of hepatic iron load measured by signal intensity ratio and R2∗ relaxometry MRI in dialysis patients. *Journal of Clinical Medicine*.

[7] Chiang H. J., Lin L. H., Li C. W. (2014). Magnetic resonance fat quantification in living donor liver transplantation. *Transplantation Proceedings*.

[8] Ji Y., Hong W., Liu M., Liang Y., Deng Y., Ma L. (2020). Intervertebral disc degeneration associated with vertebral marrow fat, assessed using quantitative magnetic resonance imaging. *Skeletal Radiology*.

[9] Hu L., Zha Y. F., Wang L. (2018). Quantitative evaluation of vertebral microvascular permeability and fat fraction in alloxan-induced diabetic rabbits. *Radiology*.

[10] Liau J., Shiehmorteza M., Girard O. M., Sirlin C. B., Bydder M. (2013). Evaluation of MRI fat fraction in the liver and spine pre and post SPIO infusion. *Magnetic Resonance Imaging*.

[11] Reeder S. B., Cruite I., Hamilton G., Sirlin C. B. (2011). Quantitative assessment of liver fat with magnetic resonance imaging and spectroscopy. *Journal of Magnetic Resonance Imaging*.

[12] Rajlawot K., Jiang T., Zhou J. (2021). Accuracies of chemical shift in/opposed phase and chemical shift encoded magnetic resonance imaging to detect intratumoral fat in hepatocellular carcinoma. *Journal of Magnetic Resonance Imaging*.

[13] Savio S. J., Harrison L. C., Luukkaala T. (2010). Effect of slice thickness on brain magnetic resonance image texture analysis. *Biomedical Engineering Online*.

[14] Wang Y. S., Zhang G. P., Yang X. (2020). Assessment of hepatic fat content in using quantitative ultrasound measurement of hepatic/renal ratio and hepatic echo-intensity attenuation rate. *Medical Ultrasonography*.

[15] Pei X. J., Lian Y. F., Yan Y. C. (2020). Fat fraction quantification of lumbar spine: comparison of T1-weighted two-point Dixon and single-voxel magnetic resonance spectroscopy in diagnosis of multiple myeloma. *Diagnostic and Interventional Radiology*.

[16] Eskreis-Winkler S., Corrias G., Monti S. (2018). IDEAL-IQ in an oncologic population: meeting the challenge of concomitant liver fat and liver iron. *Cancer Imaging*.

[17] Colgan T. J., Van Pay A. J., Sharma S. D., Mao L., Reeder S. B. (2020). Diurnal variation of proton density fat fraction in the liver using quantitative chemical shift encoded MRI. *Journal of Magnetic Resonance Imaging*.

[18] Bartoli M., Barat M., Dohan A. (2020). CT and MRI of pancreatic tumors: an update in the era of radiomics. *Japanese Journal of Radiology*.

[19] Hall M. E., Jordan J. H., Juncos L. A., Hundley W. G., Hall J. E. (2018). BOLD magnetic resonance imaging in nephrology. *Int J Nephrol Renovasc Dis.*.

[20] Linka K., Schäfer A., Hillgärtner M. (2019). Towards patient-specific computational modelling of articular cartilage on the basis of advanced multiparametric MRI techniques. *Scientific Reports*.

[21] Mi H., Yuan M., Suo S. (2020). Impact of different scanners and acquisition parameters on robustness of MR radiomics features based on women's cervix. *Scientific Reports*.

[22] Li C. Q., Chen W., Rosenberg J. K. (2014). Optimizing isotropic three-dimensional fast spin-echo methods for imaging the knee. *Journal of Magnetic Resonance Imaging*.

[23] Li T., Mirowitz S. A. (2003). Fast T2-weighted MR imaging: impact of variation in pulse sequence parameters on image quality and artifacts. *Magnetic Resonance Imaging*.

[24] Cheng C., Zou C., Liang C., Liu X., Zheng H. (2017). Fat-water separation using a region-growing algorithm with self-feeding phasor estimation. *Magnetic Resonance in Medicine*.

[25] Wen Z., Reeder S. B., Pineda A. R., Pelc N. J. (2008). Noise considerations of three-point water-fat separation imaging methods. *Medical Physics*.

[26] Peng H., Zou C., Cheng C. (2019). Fat-water separation based on Transition REgion Extraction (TREE). *Magnetic Resonance in Medicine*.

